The article "Machine Learning Approach for Cardiovascular Risk and Coronary Artery Calcification Score" was retracted in 2023. Reasons: signs of a paper mill; compromised peer review; unreliable results or conclusions.

# Machine Learning Approach for Cardiovascular Risk and Coronary Artery Calcification Score

**DOI:** 10.1155/2022/2632770

**Published:** 2022-06-23

**Authors:** C. R. Aditya, Naveen Chakravarthy Sattaru, Kumaraguruparan Gopal, R. Rahul, G. Chandra Shekara, Omaima Nasif, Sulaiman Ali Alharbi, S. S. Raghavan, S. Arockia Jayadhas

**Affiliations:** ^1^Department of Computer Science and Engineering, Vidyavardhaka College of Engineering, Mysuru, Karnataka 570002, India; ^2^Aurora Degree & PG College, Affiliated to Osmania University, Hyderabad, Telangana 500020, India; ^3^Department of Physiotherapy, College of Health Sciences, Gulf Medical University, Ajman 4184, UAE; ^4^Department of Mathematics, BMS College of Engineering, Bengaluru, Karnataka 560019, India; ^5^Department of Physiology, College of Medicine and King Khalid University Hospital, King Saud University, Medical City, PO Box 2925, Riyadh 11461, Saudi Arabia; ^6^Department of Botany and Microbiology, College of Science, King Saud University, PO Box 2455, Riyadh 11451, Saudi Arabia; ^7^Department of Microbiology, University of Texas Health and Science Center at Tyler, Tyler 75703, TX, USA; ^8^Department of EECE, St. Joseph University, Dar es Salaam, Tanzania

## Abstract

Coronary artery calcification (CAC) could assist in the discovery of new risk elements for coronary artery disorder. CAC evaluation, on the other hand, is difficult due to the wide range of CAC in the populations. As a reason, evaluating and analysing data among research have become complicated. In the Research of Inherited Risk Factors for Coronary Atherosclerosis, we used CAC information to test the effects of different analytical methodologies on the correlation with recognized cardiovascular risk elements in asymptomatic patients. Cardiac computed tomography (CT) is also seeing an increase in examinations, and machine learning (ML) could assist with the growing amount of extracted data. Furthermore, there are other sectors in cardiac CT where machine learning could be crucial, including coronary calcium scoring, perfusion, and CT angiography. The establishment of risk evaluation algorithms based on information from CAC utilizing machine learning could assist in the categorization of patients undergoing cardiovascular into distinct risk groups and effectively adapt their treatments to their unique situations. Our findings imply that for forecasting CVD occurrences in asymptomatic people, age-sex segmentation by CAC percentile rank is as effective as absolute CAC scoring. Longitudinal population-based investigations are currently underway and would offer further definitive findings. While machine learning is a strong technology with a lot of possibilities, its implementations in the domain of cardiac CAC are generally in the early stages of development and are not currently commonly accessible in medical practise because of the requirement for substantial verification. Enhanced machine learning will, however, have a significant effect on cardiovascular and coronary artery calcification in the upcoming years.

The article "Machine Learning Approach for Cardiovascular Risk and Coronary Artery Calcification Score" was retracted in 2023. Reasons: signs of a paper mill; compromised peer review; unreliable results or conclusions.

## 1. Introduction

Coronary artery disorder (CAD) is the world's leading cause of death today [1]. Clinical characteristics including angina, myocardial infarction, or unexpected deaths owing to coronary artery occlusion are the most corporate signs of CAD. Considering the intensity of these early disorder signs, a significant study objective has been to detect asymptomatic persons at risk of coronary atherosclerosis so that therapy could begin when they approach the clinical horizons. Moreover, since most noninvasive techniques of coronary atherosclerosis identification (including the treadmill activity testing or thallium scintigraphy) have limited sensitivities in younger, asymptomatic persons, earlier treatment of asymptomatic patients has proved problematic [2]. Calcium depositions in coronary arteries have been linked to atherosclerotic plaques for several decades [3, 4].

Numerous investigations ([5–7] have established durable links between CAD and the occurrence of coronary artery calcification (CAC), which can be detected by fluoroscopy, autopsy, or computed tomography (CT). Furthermore, techniques for detecting CAC using electron beam CT have been established. CAC is a more sensing marker for coronary atherosclerosis than some other noninvasive procedures, according to previous research [8, 9], and its existence predicted prospective CAD mortality and morbidity in symptomatic and asymptomatic [10] individuals. Genetics has become a significant target of study into the origins and predictions of prevalent human disorders such as CAD over the last ten decades. One area of investigation has been to learn more regarding the genetic roots of prevalent disorders, which should let us concentrate on intermediary physiological and biochemical features that can be utilized to identify people who are at risk or provide targets for earlier disorder prevention.

A secondary emphasis has been on discovering genetic changes linked to interindividual heterogeneity in illness onset, medical severity, or progression which could offer more effective disorder forecasting than these intermediary features. Even though (a) a person's genotype is more steady over a period than intermediate traits, (b) a person's genotype is not impacted by the disorder procedures, and (c) also, every gene could have impacts on numerous intermediate attributes, genotypes at loci that impact interindividual variability in intermediate attributes and are hypothesised to participate to CAD susceptibility, including the one coding for apolipoprotein E (ApoE), which could be greater predictors of risk than intermediate traits. On another side, it is worth noting that a genotype's impact on intermediary features and disorder vulnerability might shift during the course of a person's life. The impact of a genotype might well be influenced by the disorder procedure directly, or the genotypes might impact distinct collections of features or disorder resulting in various situations and at various periods.

The article "Machine Learning Approach for Cardiovascular Risk and Coronary Artery Calcification Score" was retracted in 2023. Reasons: signs of a paper mill; compromised peer review; unreliable results or conclusions.

For disorders with single-gene origins, where the mappings among genetic variability and disorder present are anticipated to be ≈1 : 1, genetic knowledge is anticipated to be used to forecast disorder severity and onset, as well as to identify actions to avoid or manage conditions. Furthermore, it is unclear if genetic variation would be useful for forecasting or managing disorders in the general populations for prevalent complicated disorders including CAD. Allelic variability in certain CAD susceptibility genes is forecasted to influence variability in CAD risk that is not represented by variability in the transitional traits currently recognized, and variability in certain transitional characteristics is anticipated to collect knowledge regarding environmental impacts and allelic variability in susceptibility genes that have not yet been assessed. As a result, an essential study query in the genetics of CAD is whether knowing about genetic diversity would enhance our capacity to forecast CAD above known risk factors. This query is particularly pertinent to the objective of recognizing young, asymptomatic persons with a higher risk of coronary atherosclerosis who might advantage the highest from risk-reduction measures. ApoE is one of the well-studied CAD susceptibility genes. The ApoE gene's frequent alleles *ϵ*2, *ϵ*3, and *ϵ*4 result in six genotypes, three of which (*ϵ*3/2, *ϵ*3/3, and *ϵ*4/3) are frequent in most populations investigated. Since its relationship has variability in lipids and apolipoprotein concentrations, which are risk elements for CAD [11], ApoE genotypic knowledge is thought to give CAD risk characteristics [12]. The comparative intensity of the e4 allele has been found to be higher in high-risk populations [13], enhanced in those with CAD in several cross-sectional and case-control research [14, 15], and raised in aged men who died of CAD throughout a five-year follow-up [16]. Investigations show that ApoE is a CAD susceptible gene; other investigations have found no link among ApoE genotypes and the risk of medically characterized symptomatic CAD [17, 18].

The article "Machine Learning Approach for Cardiovascular Risk and Coronary Artery Calcification Score" was retracted in 2023. Reasons: signs of a paper mill; compromised peer review; unreliable results or conclusions.

Coronary heart disorder (CHD) occurs in families at an early age [19]. Even though conventional risk attributes with a genetic element, including hypercholesterolemia, hypertension, and diabetes, could describe several of the genetic variations of CHD, there are supplementary genetic elements that predispose to premature CHD [20], the detectors of which would then be assisted by the identification of subjects with family records of premature CHD and their heritages. Furthermore, fewer large-scale organized initiatives to recruit cohorts depending exclusively on family descriptions of early CHD have been made [21, 22]; therefore, we identified healthful people in a research called the Studies of Inherited Risk for Coronary Atherosclerosis (SIRCA) depending on a family background of early CHD. Conventional CHD risk characteristics are linked to clinical manifestations of cardiovascular problems, including angina and myocardial infarction; nevertheless, coronary atherosclerosis occurs slowly over years. Acute myocardial infarction and suddenly death account for more than half of all major cardiovascular deaths in traditionally asymptomatic people [23]. Coronary atherosclerosis has not been conveniently available for quantifiable assessment due to its protracted, asymptomatic latency phase. Numerous asymptomatic people are classified “nonaffected” in cross-sectional research, despite the fact that they might have significant subclinical coronary atherosclerosis. Noninvasively assessing and quantifying coronary atherosclerosis in the subclinical phase of the sickness could be one way to avoid these problems.

Coronary artery calcification (CAC) is a natural part of the progression of coronary atherosclerotic plaque [24] and hence provides as a particular biomarker for coronary atherosclerosis. Whereas calcification is not present in all atherosclerosis plaques, the appearance of calcification in the coronary arteries is characteristic of atherosclerotic plaque. Electron beam tomography (EBT) could be utilized to accurately recognize as well as enumerate coronary calcification, according to studies into the molecular genetics of atherosclerosis [25–27]. The amount of histologic atherosclerosis disorders on autopsy is substantially linked with coronary calcification by EBT [27]. According to certain cross-sectional evidence, coronary calcification is greater in those with symptomatic clinical coronary disorders than in people who are asymptomatic [28]. Although there is a poor correlation among calcification at a particular coronary location and angiographic stenosis at that identical location [29], the overall likelihood of getting at minimum one cardiac stenosis or something in the coronary bed is connected with the complete coronary calcification score [30]. The relationship between coronary calcification and recognized cardiovascular risk elements has yet to be studied in larger population-based cohorts or cohorts selected depending on a family background of early CHD. Conventional cardiovascular risk characteristics, as evaluated by fluoroscopy [31] or EBT, appear to have a connection with coronary calcification, according to the minimal evidence accessible. We anticipated that measuring CAC may be utilized as a sensitive, noninvasive phenotyping technique for identifying genetic variables linked to early coronary atherosclerosis. Healthy subjects were identified in SIRCA depending on family backgrounds of early CHD. The rising triglyceride concentrations were one of the greatest predictors of CAC following age and sex; nevertheless, established risk variables (including triglycerides) described fewer than 50% of the variability in CAC between patients with CAC. Conventional risk elements cannot explain most of the variabilities in coronary atherosclerosis in a cohort particularly chosen for a family background of premature CHD, according to our findings, suggesting that this methodology might also be a robust strategic technique for recognizing new genetic elements predisposed to preventing early CHD.

The article "Machine Learning Approach for Cardiovascular Risk and Coronary Artery Calcification Score" was retracted in 2023. Reasons: signs of a paper mill; compromised peer review; unreliable results or conclusions.

Machine learning (ML), a development of the century-long search for artificial intelligence (AI), has changed the overall perception of data as well as its seeming limitless possibilities for driving changes. Machine learning is a broad term that refers to a device's capacity to train on its own by detecting similarities from massive information collections. From speech recognition and emotion analytics to automated driving, spam filters, and chatbots, this topic has generated great development across the IT industries. Although machine learning is practically ubiquitous in the information technology domain, it has been slower to catch on in the healthcare domain. The environment, on the other hand, is continuously altering. The ML community is currently focusing its attention fully on hard jobs in the medical domain, prepared with fresh ML methods, increased computing capacity, and the accessibility of huge information. For instance, in radiology, in which an ML framework has been shown to be as efficient as person radiologists in establishing presumptive diagnosis, these attempts have reaped fruits. In breast cancer pathology, ML has discovered wholly novel prognostic histological characteristics. More lately, in medical cardiology, it has been demonstrated that machine learning is more effective than medical or image analysis techniques in predicting cardiovascular or all-cause death.

The article "Machine Learning Approach for Cardiovascular Risk and Coronary Artery Calcification Score" was retracted in 2023. Reasons: signs of a paper mill; compromised peer review; unreliable results or conclusions.

Overall, the possibility for machine learning to profoundly alter the manner we practise healthcare is already widely recognized. The objectives of this analysis are threefold: (i) to describe the fundamental approach used in machine learning activities for medical spectators, (ii) to illustrate several of the opportunities in which ML has achieved implementation in cardiology, and (iii) to emphasize several of the constraints for its increased use in medicine. Machine learning (ML) is a form of artificial intelligence in which algorithms are developed on the foundation of training information collections and then used to forecast newer, possibly enormous information collections without any prior training. Deep learning is a machine learning technology that makes use of artificial neural networks (ANNs). When numerous layers are used to forecast an outcome from particular inputs, these are referred to as deep neural networks (DNN).  Figure 1 shows an instance of singular neural network vs. DNN.

Coronary computed tomography angiography (CCTA) has proven to be a reliable noninvasive approach for assessing coronary artery disorder (CAD). Several researches have established that the lack of CAD on CCTA is related with a relatively minimal risk of incident cardiovascular problems, but enhanced CAD load is associated with a graded rise in cardiovascular risks [32]. The American Heart Association (AHA), American College of Cardiology (ACC), and European Society of Cardiology (ESC) all support using coronary computed tomography angiography as a main or secondary diagnostic approach in symptomatic persons with an intermediate pretest risk of developing obstructed CAD. In daily medical practise, therefore, a large number of people who undergo coronary computed tomography angiography have mild or no CAD. As a result of the increased procedure of coronary computed tomography angiography in clinical practise, the healthcare community is becoming more interested in approaches to improve patient selection with the objective of enhancing diagnosis accuracy and expense-efficiency of CCTA usage in clinical practise. In attempt to expedite patient selection for CCTA effectiveness, a current technique tried to enhance risk classification metrics. The CAD consortium medical scores and the restructured Diamond and Forrester (UDF) scores are two population-derived risk ratings that have been designed to evaluate the pretest probability of developing CAD. Although there is a mean pretest probability of 64.4 ± 32.5 percent in the PROMISE study, only 10.8 percent of participants in the coronary computed tomography angiography arm showed obstructed CAD, although there is a median pretest probability of 53.4 ± 21.5 percent in the SCOT-HEART trial. SCOT-HEART, on the other side, discovered that 25 percent of people who had CCTA had obstructed CAD. As a result, new pretest evaluation techniques are still needed to enhance patient identification for CCTA or alternative diagnostic procedures. CAC, a particular marker of coronary atherosclerosis, has been found to have increased predicting accuracy over clinical pretest probability (PTP) evaluations in symptomatic individuals when it comes to the amount and intensity of angiographically relevant CAD. In this research, we used a contemporaneous, worldwide, and multiethnic cohort of individual people undertaking coronary computed tomography angiography assessment for coronary artery disorder identification to establish a machine learning (ML) framework based on commonly accessible medical considerations to anticipate patients probable to have disruptive coronary artery disorder on coronary computed tomography angiography and to analyse its efficacy on its own and in combined application with the coronary artery calcium score (CACS) to forecast patients probable of having obstructive CAD on CCTA.

The article "Machine Learning Approach for Cardiovascular Risk and Coronary Artery Calcification Score" was retracted in 2023. Reasons: signs of a paper mill; compromised peer review; unreliable results or conclusions.

The next sections of this research are organized as follows: Section 2 mentions existing literatures, and Section 3 mentions the proposed methodology for upgraded machine learning technique and is also able to predict cardiovascular risk and coronary artery calcification scores as well as the framework's workflow in detail.  Section 4 covers the experimental results, including data and graphs comparing them to previous studies; also, Section 5 describes discussion. Finally, Section 6 brings the research to a close.

## 2. Related Works

In [33], coronary artery calcification (CAC) could assist in the discovery of new risk characteristics for coronary artery disorder. CAC testing, on the other hand, is difficult due to the wide dispersion of CAC in the populations. As a consequence, evaluating data among research had become complicated. In the Research of Inherited Risk Variables for Coronary Atherosclerosis, they used CAC information to test the effect of different analytical methodologies on the correlation with recognized cardiovascular risk elements in 914 asymptomatic patients. (1) Linear regression of several translations of CAC ratings, (2) logistic regression utilizing CAC zero as a cut-off point, (3) Tobit regression of the log of (CAC + 1), and (4) ascending logistic regression utilizing CAC subcategories were among the multivariate assessments performed. CAC zero cut-off point logistic regression and nonlinear analysis of log CAC scores are unable to reveal relationships with certain risk elements. Ordinal regression of CAC classifications and linear and Tobit regression of the log (CAC + 1), on the other hand, revealed more connections and offered significant findings. CAC assessment approaches that are often used might miss connections with cardiovascular risk variables. They describe analytical procedures that are expected to produce continuous findings and suggest using at minimum two different multivariate techniques.

The article "Machine Learning Approach for Cardiovascular Risk and Coronary Artery Calcification Score" was retracted in 2023. Reasons: signs of a paper mill; compromised peer review; unreliable results or conclusions.

In [34], the endothelium's soluble epoxide hydrolase (sEH) regulates endogenous epoxide concentrations, which is an essential component in cardiovascular functioning control. The researchers looked at the link among frequent operational polymorphisms in the individual coronary artery calcification (CAC) and sEH gene in younger, mostly asymptomatic non-Hispanic white and African-American people. The link among the sEH Arg287Gln polymorphisms and the existence and amount of CAC was studied using multivariable Tobit regression and logistic regression techniques. Simulations were generated that took into account races (excluding racial group analysis), smoking, age, sex, BMI, LDL cholesterol, HDL cholesterol, and systolic BP. The frequency distribution of alleles and genotypes was not substantially varied among the two ethnicity categories (*P* = 0.33 as well as *P* = 0.28, correspondingly). In African-American subjects, the Arg287Gln polymorphisms of the sEH gene had been a substantial prediction of the CAC state, whether independently or after correcting for several other risk components. African-American participants who carried at minimum one copy of the Gln287 allele had a twofold higher hazard of coronary artery calcification than those who did not (96 percent CI, 2.2 to 3.1; *P* = 0.03). In white participants, there was no link among the Arg287Gln polymorphisms and the likelihood of developing CAC (OR, 0.9; 96 percent CI, 0.5 to 1.3; *P* = 0.49). The results of multivariate Tobit modelling were comparable to those of logistic regression modelling, demonstrating that the Arg287Gln polymorphisms represented a significant individual prediction of CAC occurrence and quantity in African-Americans but not in whites. These findings point to a fascinating and potentially unique involvement for sEH in the aetiology of atherosclerosis that warrants further exploration.

In [35], there have been significant changes in the risks of cardiovascular disorder (CVD) occurrences correlated with coronary artery calcium (CAC). Compared to quartiles of actual CAC scoring, they assessed the link of the coronary calcium quartile to CVD incidents using age-sex cut lines from a wide dataset of asymptomatic people as a feasible standardized approach for documenting incident risks connected with CAC. They used age/sex-based cut factors on 928 asymptomatic women and men (median ages 54 decades) that were monitored for a median of 3.3 years and had 28 CVD incidents validated throughout that time. With and without age/sex stratification, Cox modelling was utilized to assess the relationship between the quartiles as well as the hazard of developing CVD incidents. The number of incidents (and percentage occurrence) in the first, second, third, and fourth quartiles of coronary calcification was  13 (6.4%), 2 (2.0%), 4 (0.9%), and 9 (4.5%), for the age and sex stratified quartiles (*P* = 0.001), and 4 (1.0%), 0 (0%), 7 (3.0%), and 17 (7.3%) for the actual scoring quartiles (*P* = 0.001). There was a moderate increase in CVD occurrences between individuals in the third quartile (related risks (RR) 4.3, *P* = 0.02) in multivariate analyses controlled for many other risk variables, with a higher risk identified between those in the fourth quartile (RR 6.0, *P* < 0.01) (contrasted with the first quartile). The results were similar when using actual CAC assessments, with RR = 2.6 (*P* = 0.14) for the third quartile and RR = 6.4 (*P* < 0.01) for the fourth. Their findings imply that for forecasting CVD occurrences in asymptomatic people, age and sex stratification by CAC percentile ranking is as precise as actual CAC scorings. Longitudinal population-dependent investigations are currently underway and would offer further definitive findings.

The article "Machine Learning Approach for Cardiovascular Risk and Coronary Artery Calcification Score" was retracted in 2023. Reasons: signs of a paper mill; compromised peer review; unreliable results or conclusions.

In [36], coronary computed tomography angiography (CCTA) is a medically validated as well as effective approach for assessing coronary artery disorder. The fractional flow reserve (FFR) could be considered using coronary computed tomography angiography information collections as CT-FFR. Although contrasted to conventional fractional flow reserve in earlier tests, this approach has shown to be effective in diagnosing lesion-specific ischemia. Recent research has revealed a number of advantages, such as better treatment recommendations to effectively explain the maintenance of individuals with suspicious coronary artery disorder, better outcomes, and lower medical expenditures. A technological technique to CT-fractional flow reserve computation employing an artificial intelligence (AI) deep machine learning (ML) technique has just been developed. Compared to coronary computed tomography angiography, machine learning techniques present knowledge in a rather consistent, repeatable, and reasonable method, with increased diagnosis precision. The technological basis, medical verification, and deployment of machine learning implementations in CT-FFR are all covered in this paper.

The article "Machine Learning Approach for Cardiovascular Risk and Coronary Artery Calcification Score" was retracted in 2023. Reasons: signs of a paper mill; compromised peer review; unreliable results or conclusions.

In [37], the noninvasive assessment of coronary atherosclerosis uses electron beam CT (EBCT) measurement of coronary artery calcification (CAC). They conducted a follow-up trial to see if CAC extent, as evaluated by EBCT during angiography, is associated with future severe cardiovascular occurrences, such as cardiac mortality and nonfatal myocardial infarction (MI). Selective coronary artery disorder (CAD) risk variables, past CAD occurrence histories (revascularization or MI), and angiographic results (number of infected arteries and total disorder burden) were also evaluated for their ability to forecast subsequent severe occurrences. For an average of 6.9 years, 238 individuals who underwent simultaneous EBCT imaging and coronary angiography were approached. Throughout the follow-up, the vital situation and histories of MI were established. To examine the predicting potential of coronary artery calcification extension with specified coronary artery disorder hazard variables, coronary artery disorder incident histories, and angiographic results, Cox proportionate risks algorithms were utilized. The average coronary artery calcification scoring was 160 (range from 0 to 7633). The 22 individuals who had difficult episodes throughout follow-up were senior and had much more coronary artery calcification and angiographic illness (*P* < 0.05). Throughout the follow-up, only 1 of 87 individuals with a CAC scoring of <20 had a future hard incident. Patients with CAC scores less than 100 had a considerably higher chance of surviving an event than those with scores more than 100 (comparative hazard 3.20; 95 percent CI 1.17 to 8.71). Both age and CAC extensiveness estimated severe occurrences in a stepwise multivariate analysis (risk factors 1.72 and 1.88, correspondingly; *P* < 0.05). Coronary artery calcification range on electron beam CT intensely predicted upcoming hard cardiovascular incidents in individuals having angiography and contributes significant prognostic knowledge.

From [38], insulin resistance syndrome, which includes insulin resistance as well as a number of metabolic disorders, is linked to a higher hazard of symptomatic coronary artery disorder. Asymptomatic people with more coronary calcification have more coronary plaques and are more possible to suffer a heart attack or stroke in the prospective. In 1160 asymptomatic women and men, coronary artery calcification scoring, anthropometric and metabolic characteristics, and fasted and stimulating glucose and insulin concentration levels were assessed using electron beam computed tomography. Homeostasis, glucose, and insulin prototype evaluation (HOMA) insulin sensitivity was strongly linked with coronary artery calcium scoring. Calcium scores were considerably connected with HDL and periphery fats and considerably associated with age, overall high cholesterol-density lipoprotein (HDL) ratios, intra-abdominal adiposity, lower-density lipoprotein, BP, HOMA beta cell activity, and triglycerides. Excluding two hours of glucose, these relationships persisted important for those patients with fasting serum glucose 126 mg/dL or fasting blood glucose 110 mg/dL. Age, sex, family background of early intra-abdominal obesity, lower-density lipoprotein, coronary artery disorder, and smoking are all associated with calcification scoring in a multivariable assessment. Coronary artery calcium scoring was not significantly linked with HOMA insulin resistance, HDL, glucose, triglycerides, insulin, blood pressure, or beta cell activity. People with insulin resistance who are asymptomatic have high coronary calcium assessments. With poor glucose tolerance and regular fasting serum glycolysis, the link between insulin resistance and coronary calcification remains. Especially in asymptomatic nondiabetic people, central/visceral obesity might be a predictor of insulin resistance and atherosclerosis.

The article "Machine Learning Approach for Cardiovascular Risk and Coronary Artery Calcification Score" was retracted in 2023. Reasons: signs of a paper mill; compromised peer review; unreliable results or conclusions.

In [39], the goal of that research was to see how the coronary artery calcium (CAC) scores affected the diagnostic effectiveness of coronary computed tomography (CT) angiography (CCTA) resultant component flow reserve calculated using machine learning (CT-FFR). CT-FFR is a consistent methodology for identifying ischemia in particular lesions. New CT-FFR procedures based on machine learning artificial intelligence approaches are quick and do not demand as much computationally fluid dynamics. The impact of the CAC scores on the machine learning technique's diagnostic effectiveness is still to be examined. The MACHINE (Machine Learning Predicated CT Angiography Determined FFR: A Multicenter Registry) registry information was used to study 482 arteries from 314 patients (62.3 ± 9.3 years, 77 percent male) who underwent coronary computed tomography angiography accompanied by invasive FFR. The Agatston technique was used to calculate CAC scoring. On a per-vessel source, the diagnostic effectiveness of CT-FFR in detecting lesion-specific ischemia was evaluated using conventional FFR as the reference standard throughout every Agatston score classification (CAC 0, >0 to < 100, 100 to < 400, and ≥ 400). In CAC, machine learning-dependent CT-FFR performed better than coronary computed tomography angiography individually, with a considerable variation in CT-FFR effectiveness as calcification burden/Agatston calcium scoring improved.

The article "Machine Learning Approach for Cardiovascular Risk and Coronary Artery Calcification Score" was retracted in 2023. Reasons: signs of a paper mill; compromised peer review; unreliable results or conclusions.

In [40], to regulate the arrangement and consistency of entirely computerized coronary artery calcium (CAC) scoring in people who are screened for lung cancer, a low-dose chest CT scan was examined (noncontrast improved, nongated). To build a typical reference for coronary artery calcification, an early implementation of a system utilizing a coronary calcium atlas and machine learning technique was used to provide automated calcium scoring. Every scanning was then examined by one of four professional raters. Whenever necessary, the raters made corrections to the findings that had been discovered by automaticity. Furthermore, an impartial observer reviewed the individually modified findings and excluded images with significant segmented mistakes. Following that, a completely automated coronary calcium scoring system was used. The number of calcifications, the Agatston score, and the CAC volumes were all calculated. The percentages of the agreement were calculated, and Bland-Altman plots were examined to evaluate consistency. The linearly weighted kappa (*k*) for Agatston strata and the intraclass correlation coefficient (ICC) for continuous data were used to measure reliability. Metal artefacts or gross segmented problems resulted in the exclusion of 44 images (2.5%). The autonomous scoring for the remaining 1749 scans showed a median Agatston scoring of 39.6 (*P*25–*P*75 : 0–345.9), an average volume value of 60.4 mm^3^ (*P*25–*P*75 : 0–361.4), and an average number of calcifications of 2 (*P*25–*P*75 : 0–4). Among the automation and referenced ratings, *k* showed very strong reliability (0.85) for Agatston risk groups. The Bland-Altman charts revealed automatic quantification of underestimated calcium score levels. The median variation in Agatston scoring was 2.5 (*P*25–*P*75 : 0.0–53.2), CAC volume was 7.6 (*P*25–*P*75 : 0.0–94.4), and the number of calcifications was 1 (*P*25–*P*75 : 0–5). The ICC was excellent for the Agatston scoring system (0.90), calcium volume (0.88), and frequency of calcifications (0.64). Considering an underestimation of the quantity of calcification when contrasted to comparison scores, complete automation of coronary calcification assessment in a lung cancer monitoring environment is possible with appropriate accuracy and consistency.

In [41], artificial intelligence, particularly machine learning (ML), has grown in popularity in recent decades as a result of its flexibility and promise for tackling complicated issues. Indeed, machine learning provides for the effective management of large amounts of information, enabling the resolution of previously unsolvable problems, particularly with deep learning, which employs multidimensional neural networks. Cardiac computed tomography (CT) is also seeing an increase in examinations, and machine learning (ML) could assist with the growing amount of extracted data. Furthermore, there are other sectors in cardiovascular CT where ML could be crucial, including perfusion, coronary calcium scores, and CT angiography. Image postprocessing and preprocessing, as well as the establishment of risk evaluation algorithms depending on scanning data, are two of the most common uses of machine learning. When it comes to picture preprocessing, machine learning could assist enhancement of image clarity by optimising acquiring techniques or eliminating artefacts that might make image evaluation and interpretation difficult. Image postprocessing using machine learning could assist automated categorization and reduce inspection processing durations, as well as provide instruments for tissue characterization, particularly in the case of plaques. The establishment of risk evaluation algorithms based on information from cardiac CT utilizing machine learning may assist in the categorization of patients undergoing cardiovascular CT into distinct risk groups and effectively adapt their treatments to their unique situations. Although machine learning is a strong technology with a lot of potentials, its implementations in the domain of cardiovascular CT are currently in the early stages of development and are not currently commonly accessible in medical practise because of the requirement for substantial verification. ML will, however, have a significant effect on cardiovascular CT in the coming years.

The article "Machine Learning Approach for Cardiovascular Risk and Coronary Artery Calcification Score" was retracted in 2023. Reasons: signs of a paper mill; compromised peer review; unreliable results or conclusions.

In [42], a framework of artery characteristics was constructed using machine learning to distinguish between individuals who die or have cardiovascular problems and those who do not. The results were contrasted to those of traditional scoring. Radiologists dissected coronary CT angiography into four characteristics for every one of the 16 coronary sections. Four different types of machine learning models were investigated. The coronary artery disorder reporting and data system (CAD-RADS) score was one of five traditional artery ratings used for comparisons. Coronary heart disorder deaths, every affected mortality, and nonfatal myocardial infarction coronary deaths were the results studied. The region below the receiving operational parameter curves was used to evaluate scoring effectiveness (AUC). There were 380 fatalities from various factors, 70 deaths from coronary artery disorders, and 43 nonfatal myocardial infarctions documented. For those cause mortality, the AUC for machine learning (*k*-nearest neighbours) was 0.77 (95 percent confidence duration:  0.76, 0.77) versus 0.72 (95 percent assurance period:0.72, 0.72) for CAD-RADS (*P* < 0.001). Machine learning had an AUC of 0.85 (95 percent confidence period: 0.84, 0.85) for coronary artery cardiovascular disorder fatalities against 0.79 (95 percent probability duration: 0.78, 0.80) for CAD-RADS (*P* < 0.001). In determining whether to begin statins, if the decision is produced to regard 45 patients to confirm that each patient would also die of coronary disorder later, the machine learning scoring system guarantees that 93 percent of patients with occurrences would be handled; if CAD-RADS is utilized, only 69 percent of patients with events would be handled. Machine learning approaches distinguished patients who had an unfavourable occurrence from those who did not higher than the coronary artery disorder monitoring and information framework as well as various ratings.

## 3. Proposed Methodology

Many analytical techniques utilized two multivariate parameters. The initial looked at age-adjusted relationships among risk factors and CAC. The second was fully corrected for every abovementioned risk variable. Men and women were studied individually in fully adjusted algorithms to see if there were any sex-specific correlations among pairings of hazard components. In completely multivariate assessments which comprised both men and women, correlations among sex and hazard variables were established. The probability proportion analyses were used to determine the importance of connections. We employed bootstrap approaches (1000 iterations) to generate durable 96 percent confident ranges (96 percent CI) for point estimations across various approaches since the distributions of CAC and its modifications, particularly ln(CAC + 1), were not normal. The Brant testing was used to evaluate the proportionate odds assumptions of ordinal analysis.

Fifty variables were accessible for study (25 clinical, 20 laboratory, and 5 CACS variables). Automatic feature identification, a randomized partition of the derived cohort into a training (65 percent of information) and testing (35 percent) set, and modelling development with an enhanced ensemble technique (LogitBoost) were all part of the machine learning process (Figure 2). The open-source Waikato Environment for Information Assessment framework was used to deploy machine learning algorithms. There were 44 CCTA variables and 20 medical characteristics to choose from (Figure 2). For the overall procedure, machine learning included automatic component selection based on data gained ranking, modelling development using an enhanced ensemble technique, and 10-fold stratified cross-validation (Figure 2) [43]. The open-source Waikato Environment for Information Assessment framework was used to deploy machine learning algorithms.

The article "Machine Learning Approach for Cardiovascular Risk and Coronary Artery Calcification Score" was retracted in 2023. Reasons: signs of a paper mill; compromised peer review; unreliable results or conclusions.

### 3.1. Data Collection

After the recruitment process, individuals' race, sex, and age were self-reported and confirmed during the baseline clinical session. With the individual dressed in light clothing and no shoes, body weight was estimated to the closest 0.2 pounds on calibrated scales. A vertical ruler was used to estimate heights to the nearest 0.5 cm. The BMI was evaluated as weight (kg) divided by height (m^2^). The Friedewald formula was employed to determine LDL cholesterol. With the individual seated but after a 5-minute pause, blood pressures were monitored on the right arm with a random-zero sphygmomanometer at every assessment. Phases 1 and phases 5 Korotkoff noises were used to measure systolic and diastolic pressures. At 1-minute durations, three assessments were obtained. The BP reading was calculated as the average of the second and third assessments. The tobacco consumption of individuals was determined using a CARDIA-specific tobacco questionnaire. The processes for information collection were recently discussed in detail.

Coronary calcium was assessed using a CT scan of the chest at the year-15 assessment. In two successive scans, 40 continuous 2.5 to 3 mm thick transverse pictures from the roots of the artery to the apex of the heart were obtained using electron beam computed tomography and multiple detector computed tomography scanning. Individuals were examined over a hydroxy-apatite phantom to enable picture noise and brightness scanning as well as adjustment for scanning variances. The results of both scannings were sent digitally to the CARDIA computed tomography reading center, where a qualified cardiovascular radiologist reviewed every picture and used specifically created image processing technology to identify probable foci of coronary calcification. For every calcification lesion, a calcium rating was generated by multiplying the focus' region by a measurement depending on the highest CT value in the concentration. This measurement varied from 1 to 4, with 1 = 131 to 200 HU, 2 = 201 to 300 HU, 3 = 301 to 400 HU, and 4 = 401 or more HU. The overall calcium rating for the individual was calculated by adding any lesion within a specific artery throughout all arteries. An expert investigator without an understanding of the scanning results assessed every scanning sets with at least one nonzero result and a randomized sampling of those with a 0 score to validate the absence or presence of coronary calcium. CAC statistics were gathered on 1500 people, with 1205 of them having DNA samples.

The article "Machine Learning Approach for Cardiovascular Risk and Coronary Artery Calcification Score" was retracted in 2023. Reasons: signs of a paper mill; compromised peer review; unreliable results or conclusions.

### 3.2. Measurement of CAC

CAC was determined utilizing a standardized methodology on an Imatron C-150 electron beam computerized tomography scanner. Coronary artery calcification was characterized as a hyperattenuating concentration in coronary arteries that was at minimum four contiguous pixels in dimension (— in other words, 1.04 m m^2^) and had radiographic attenuated coefficients (computed tomography score) greater than 130 Hounsfield units throughout. Every tomogram was reviewed for technological reliability and scored consistency by established radiologists, who then evaluated the results. The CAC scores established were used to determine the quantity of CAC. Participants with detected coronary artery calcification and coronary artery calcification levels ≥ 70th percentile for their sex and age depending on coronary artery calcification scores from a community-based sampling of asymptomatic people without hazard characteristics were defined as having a significant coronary artery calcification burden and contrasted to those with coronary artery calcification values < 70th percentile. The 70th percentile indicates those who are thought to be the most at risk for a prospective occurrence.

### 3.3. Coronary Calcium Sample

We used cardiac gating CT to quantify coronary vascular calcification in two ARIC fields' centers. In previous ARIC case-control investigations, the targeted samples contained two categories that had been thoroughly defined for nonconventional risk variables. Every monochrome subject with no medical cardiovascular illness by visit 2 and “higher” average carotid IMT (greater than 1 mm for whites, greater than 0.946 mm for blacks) in ultrasounds from visits 1 and 2 were combined in one group (ultrasound instances). The second category (randomized category) consisted of a stratified random sample of black and white people who had carotid IMT information but no clinical cardiovascular illness. Within two age gender, strata, and two carotid IMT classifications (“low” = mean IMT < 0.787 mm as well as “medium” = mean IMT ≥ 0.787 but no ultrasonography instance), various sampling probabilities were employed to choose for the randomized groups. Computation of *z* using the inputs *x*_*i*_:

(1) $$\begin{array}{c} z=\underset{i}{\sum }\omega_{i}*x_{i}+b. \end{array}$$

Using *z*, compute *a*, which is equivalent to *y* at the output layer:

(2) $$\begin{array}{c} a=\psi \left(z\right). \end{array}$$

*ω*_*i*_ are the weights, *b* is the bias, and *ψ* is said to be the activation function. The remaining patients were called and given a screening questionnaire to rule out anyone with a recognized CHD, recently substantial radiation, or some other conditions that could have hampered CT interpretations (including metal prostheses or severe obesity in the spine). The CT test was accomplished by 48 percent of the 459 Forsyth individuals (*n* = 279), 20 percent were removed, deceased, or no more residing in the region, and 32 percent were rejected. These proportions were 51 percent (*n* = 203), 32 percent, and 38 percent, respectively, of the 373 people who were searched in Minneapolis. Finally, 32 percent (*n* = 89) of ultrasound instances and 56 percent (*n* = 393) of the randomized category accomplished the cardiac CT test. As a result, the coronary calcium samples consisted of volunteers who did not have a clinically diagnosed CHD. Nonetheless, their parameters were not significantly dissimilar from those of the entire ARIC research (Table 1) [44], with the most notable variations being thicker carotid IMT, lower diabetes, and lower hypertension.

The article "Machine Learning Approach for Cardiovascular Risk and Coronary Artery Calcification Score" was retracted in 2023. Reasons: signs of a paper mill; compromised peer review; unreliable results or conclusions.

### 3.4. Coronary Calcium Assessment

We used cardiac gating mechanically or helical CT to quantify coronary calcium. A single-slice helical CT device with retrospective cardiac gating was used at the Forsyth center (generalized electrical healthcare devices, CTi, Milwaukee, WI). The gantry rotational duration on this device is 800 milliseconds, and the imaging temporal resolution is 533 milliseconds per picture. A 4-slice CT scanner with anticipated progressive cardiac triggering was utilized in the Minnesota field center. The gantry rotation duration on this device is 500 milliseconds, and the image temporal resolution is 250 milliseconds for each image. On the Siemens device, slice thickness was 2.5 mm, but on the GE framework, it was 3 mm. Both devices employed the partial scanned reconstructing technique and the conventional reconstructed kernel.

A calcium phantom (image classification) was used for every cardiac CT exam. Individuals were educated on how to retain their breathing before being positioned supine on the CT couch. The chest was fitted with electrocardiogram leads. Two simulated cardiac gated scannings were obtained through the heart following the early scouting photos. The starting point was 2 cm beyond the carina, and the complete heart was photographed in a single breath hold of 25 to 45 seconds. (The individual's pulse rate and the duration of the heart across the *z*-axis determine the individual's breath hold duration.) For coronary calcification assessment, the CT pictures were connected to a computing workspace. For every repeat scan, a typical Agatston scoring was generated, with calcification defined as two consecutive pixels of 241 HU. In Forsyth County, scoring was done using the SmartScore programme on a GE Advantage Windows computer. Scoring was done on a Siemens Virtuoso workstation in Minnesota. (A correcting element of 2.5/3.0 was given to the calcification score because this application expected a 3 mm slice thickness.) Every research was examined by a board-certified radiologist (AS or JC) to ensure the accuracy of the calcification measurement and to identify any ancillary abnormalities. For evaluation, the two replicated calcification scores were averaged because they were strongly linked (*r* = 0.97 for Minneapolis, Spearman *r* = 0.98 for Forsyth County).

The article "Machine Learning Approach for Cardiovascular Risk and Coronary Artery Calcification Score" was retracted in 2023. Reasons: signs of a paper mill; compromised peer review; unreliable results or conclusions.

### 3.5. SNP Genotyping

Lipid metabolism, inflammation, ion transport, renin-angiotensin system, and vascular wall biology were chosen as biological processes or positioning candidate genes from networks recognized to be related to CAD as well as hypertension. SNP genotyping was performed on the Sequenom MassARRAY System with a mass spectrometer-based detecting framework and an ABI Prism Sequential Detecting Device with a fluorogenic TaqMan assay. The researchers can provide primers and probing sequence data upon demand.

### 3.6. Quality-Control Program

The 96 percent bounds of agreements were utilized as a portion of a reliability procedure to detect dual scan run outcomes in individuals that were surprisingly dissimilar and to discover the explanation for the differential. A radiologist (PFS) reviewed the outcomes of 35 dual scan runs in which the arithmetical variances were beyond the 96 percent bounds of agreement. Triggering difficulties, gaps, partial quantity impacts, overlaps, arrhythmias, heart or patient movement, ECG misregistrations, table incrementation, errors in patient positioning, noise, artefact, aortic rim, foci not in an artery, and pericardial calcifications or valvular were all scrutinised in these findings.

### 3.7. CAC Variation across Time

A scattering plot of the median calcific region in the dual scanning tests at follow-up versus the calcific region in the singular scanner test at baseline was created using information from the individuals who had a singular scanning test at baseline and double scanning tests at follow-up. Lines reflecting the spectrum of calcification region anticipated from the 96 percent ranges of agreements for the 1000 individuals were superimposed on the plot. The person was regarded to have no changes in the identifiable quantities of CAC if the baseline outcome was within the expected limit of the follow-up findings. The person was judged to show improvement in the identifiable proportion of CAC if the baseline results were to the left of the expected limit at follow-up. That is, the baseline outcome in the double scanning tests at follow-up was significantly lower than the median. The person was judged to have regression in the identifiable level of CAC if the preliminary outcome was to the right of the anticipated limit at follow-up. That is, the baseline results in the double scanning tests at follow-up were significantly higher than the median.

The article "Machine Learning Approach for Cardiovascular Risk and Coronary Artery Calcification Score" was retracted in 2023. Reasons: signs of a paper mill; compromised peer review; unreliable results or conclusions.

## 4. Evaluation of Risk Factors

After an overnight fast, high-density lipoprotein cholesterol (HDL-C), overall cholesterol, and triglycerides are restrained utilizing established enzymatic techniques. The glucose oxidase technique was used to determine plasma glucose levels. The Friedwald methods were used to determine low-density lipoprotein cholesterol. Weight/height^2^(kg/m^2^) were employed to determine the body mass index (BMI):

(3) $$\begin{array}{c} \text{BMI}=\frac{\text{mass }\left(\text{kg}\right)}{\text{height }\left({\text{m}}^{2}\right)}. \end{array}$$

A random-zero sphygmomanometer was employed to assess the diastolic and systolic blood pressure readings in the right arm. The median of the 2nd and 3rd estimations was assessed after three assessments collected at a minimum of 2 minutes apart. The Clauss (clotting time-based) technique was used to detect fibrinogen, and an extremely effective immunoturbidimetric test was used to evaluate C-reactive protein. Polyacrylamide gel electrophoresis was used to determine the particulate sizes of low-density lipoproteins. As recently mentioned, plasma homocysteine was determined utilizing a liquid chromatography-electrospray tandem mass spectrometry technique. The SPQTM Testing Instrument was used to assess *Lp*(*a*) in serum by employing an immunoturbidimetric assay [45].

### 4.1. Analytical Statistics

In total, 1000 people were tested to see if the double scanning tests were repeatable (at follow-up, 80 people had double scans, while 785 had double scans at the start). The Mc-Nemar testing was utilized to assess the equalization of CAC prevalence in scanning sessions 1 and 2 for comparability with other research outcomes on the reliability of double scanning exams for CAC. To eliminate skewness, the regular logs (ln[calcific area + 1]) were used to modify the calcific region in every scanning session. In scanning runs 1 and 2, a paired *t* testing was utilized to see if the mean converted calcific region was the same. To measure the correlation among translated calcific regions in the dual scanning tests, the intraclass association coefficients were determined. The nontransformed calcific region discrepancies among the dual scanning tests were shown arithmetically and compared to the median calcific region.

The article "Machine Learning Approach for Cardiovascular Risk and Coronary Artery Calcification Score" was retracted in 2023. Reasons: signs of a paper mill; compromised peer review; unreliable results or conclusions.

The consistency of assessment outcomes was assessed using the regression approach for nonuniform distribution variances. In a nutshell, we utilized linear regression to describe the arithmetic differential *D* as a proportion of the median calcific region *A*, using the equations

(4) $$\begin{array}{c} D=b_{0}+b_{1}A, \end{array}$$

where *b*_0_ is the intercept and *b*_1_ is the slopes of the linear regression line. The dispersion of the absolute values of the residual *R* from the preceding modelling as a consequence of the median calcific region was then modelled using linear regression with the formula *R* = *c*_0_ + *c*_1_*A*, where *c*_0_ is the interception and *c*_1_ is the slopes of the linear regression line. The 96 percent bounds of agreement were derived by integrating the variable estimations from both of these approaches:

(5) $$\begin{array}{c} b_{0}+b_{1}A\pm 3.57\left(c_{0}+c_{1}A\right). \end{array}$$

We utilized 3.57 instead of 1.97 in this formula since we were modelling the actual significance of the residuals instead of the residuals altogether. The actual values of the residuals would follow a half-normal distribution, therefore multiplying 1.97 by *π*/2 to get the exact values. The 96 percent ranges of agreements and arithmetical variances were shown against the mean calcification region. We calculated the calcific region anticipated at the upper and lower 96 percent ranges of agreement for double scanning tests with a specific median utilizing these boundaries of agreement. Findings acquired minutes or decades apart were compared using knowledge from these limitations.

### 4.2. Experimental Results

The prevalence of coronary, peripheral and cerebral, and vascular disorders in the research participants was significantly associated with coronary artery calcium scores. The pervasiveness of ASVD is shown in Figure 3 by the calcium score group.  Table 2 shows the percentage of participants having vascular disorders in every calcium score level.

### 4.3. Coronary Artery Calcification

Table 3 shows the incidence of coronary artery calcification and average calcium readings in healthy restrictions and patients with earlier stage and developed RA. Patients with developed RA had a mean coronary artery calcium score of 41.3 (IQR 0–369.9), contrasted to 0 (IQR 0–53.7) in those with earlier disorder and 0 (IQR 0–20.3) in controls (*P* = 0.002). Individuals with developed RA (60.5%) had greater coronary artery calcification than those with earlier RA (53.2%) or regulate (49.5%) (total *P* = 0.017, individuals with earlier RA contrasted to controls *P* = 0.68, individuals with developed RA contrasted to involves *P* = 0.007).  Figure 4 shows the pervasiveness of coronary artery calcification in restrictions and patients with RA based on age groups of fewer than 50 years, 50–59 years, 60 years, and older. The association between age and illness condition was considerable (*P* < 0.06 for interactions). The pervasiveness of coronary artery calcification was higher in patients with documented RA compared to regulate system at ages < 50 and 50–59 years (also *P* < 0.06), while the differential was not significant across subgroups of people aged ≥60 years.

The article "Machine Learning Approach for Cardiovascular Risk and Coronary Artery Calcification Score" was retracted in 2023. Reasons: signs of a paper mill; compromised peer review; unreliable results or conclusions.

### 4.4. The Association between Individuals' Illness Features and Coronary Artery Calcification

Individuals with earlier time RA and those with developed RA have different clinical features (Table 4). Individuals with existing RA had higher cumulative exposure to drugs used to manage the condition, as anticipated. On the DAS28, individuals with early and advanced RA had equivalent evaluations of disorder activities, whereas patients with advanced illness had greater M-HAQ scores (*P* = 0.03) and ESRs (*P* = 0.05). Patients with earlier stage RA had a mean swollen joint count of 5.0 ± 5.7, while those with advanced RA had a mean swollen joint count of 5.2 ± 5.6. In both categories, about 18 percent of individuals were getting tumour necrosis component blocking therapy. Table 4 shows the features of RA patients established on the degree of coronary artery calcification (moderate-to-severe, none, and mild). In unadjusted assessments, RA patients with coronary artery calcification had greater higher systolic BP, age, male sex, increased homocysteine concentration levels, greater overall pack-years of smoking, and greater ESR. Only pack-years of smoking (OR 2.03, *P* = 0.05) and greater ESR (OR 2.03, *P* = 0.06) remain substantially linked with intense coronary artery calcification in individuals with RA after controlling for sex and age as shown in the graph in Figure 5.

## 5. Discussion

Coronary artery disorder is a frequent disorder that is connected with a high rate of mortality, medical costs, and morbidity. Over the decades, it has been standard practise in medical practise to use proven diagnosis modelling of the PTP of persistent, but obstructed, CAD to guide downstream assessment. The majority of existing algorithms performed poorly (with notable overestimation of risk in specific categories, including women), and there are limited investigations on the impact of PTP-based algorithms on medical decision about further verification or patient results. As a consequence, medically oriented algorithms could forecast the PTP of consistent CAD and so serve as gatekeepers to identifying low-risk participants who are anticipated to have obstruction coronary artery disorder and therefore do not require additional diagnostics assessment to be needed. We used easily accessible medical characterization in wide multiple locations; multiethnic populations undergo medically warranted CCTA for the diagnosis of coronary artery disorder in the current study. We used machine learning (ML) as a unique analytical method that is optimised for the production of efficient predicting algorithms and discovered that the generated ML algorithm accurately forecasts the prevalence of obstructed CAD on CCTA, particularly in younger people with atypical characteristics. In addition, suitable calibration, increased categorization, and superior discrimination of nonevents were discovered. The use of a machine learning algorithm in a healthcare context may assist to automate the procedure of identifying suitable individuals for any further diagnostic examination while avoiding more time-consuming regular medical tasks.

The article "Machine Learning Approach for Cardiovascular Risk and Coronary Artery Calcification Score" was retracted in 2023. Reasons: signs of a paper mill; compromised peer review; unreliable results or conclusions.

Diagnostic scanning techniques are routinely used in excess. As a consequence, risk classification and PTP evaluation have become more important before the start of downstream analysis. In addition to preventing unnecessary investigations, the ESC suggests using the CAD consortium medical scores, whereas the ACC/AHA suggests using the Duke Clinical Score (DCS) or UDF as a component of the medical evaluation of the PTP with probable consistent coronary artery disorder. Furthermore, several studies have revealed that some risk evaluation algorithms work poorly in some groups. Furthermore, various algorithms have been confirmed in multiple exterior populations, with a recent tendency towards weaker discriminative capacity. Variations in derivation (use of diverse scanning techniques and also varied cut-off levels for defining obstructing CAD, use of imputation approaches for lacking results, etc.), modelling complexities, and uneven external verification are all factors that restrict their use in everyday practise. There is a demand for complete simulations that develop through the duration of an ever-varying situation where individuals are longitudinally developing as a consequence of altering eating patterns, primordial, preventive activities, and environmental exposures. To this goal, machine learning is rapidly being used in the cardiovascular field. Machine learning entails techniques that are particularly designed to uncover relationships among information that go beyond the present one-dimensional statistical methodologies. Furthermore, machine learning makes use of the growing accessibility of computing energy and memory capacity to give immediate results. In a period of accuracy treatment, machine learning offers the ideal chance to utilize the progressively complicated information that is accessible whereas enhancing forecasting. Furthermore, machine learning has demonstrated to be a far more potent instrument for forecasting in a variety of cardiovascular implementations.

The article "Machine Learning Approach for Cardiovascular Risk and Coronary Artery Calcification Score" was retracted in 2023. Reasons: signs of a paper mill; compromised peer review; unreliable results or conclusions.

The integration of CACS into predicting algorithms has already been proven to boost effectiveness; therefore, our data indicate that adding CACS to the machine learning algorithm resulted in the finest predictions. The integration of the CACS to the expanded CAD consortium medical scoring, for example, was discovered to considerably boost the C-statistic for the forecast of obstructed CAD on invasion coronary angiography from 0.79 to 0.88. In a sample of 1000 people suspicious of possessing coronary artery disorder and undergoing CCTA examination, adding the Agatston scores to the DCS enhanced the precision of forecasting of obstructed coronary artery disorder compared to the DCS alone (AUC 0.917 vs.AUC 0.825, correspondingly, *P* < 0.06). Considering the graduated and consistent association among rising CACS and the occurrence of obstructed CAD, the notion that the CACS increases the assessment of the risk of obstructed CAD is predicted. The majority of modern calcification scoring tests expose you to lower than a millisievert of radiation. The capability of the machine learning system to accurately categorize patients without obstructed CAD when combined with CACS may result in lower radiation exposures and expenditures. Furthermore, prospectively randomized tests that concentrate on evaluating the efficiency and security of such a strategy are needed to back up that conclusion [32].

## 6. Conclusion

In asymptomatic patients receiving a healthcare assessment, the forecasting methodology generated from ML techniques demonstrated a robust capacity to forecast CAD and cardiovascular risk, as well as superior recategorization over known traditional risk forecasting methodologies.

- Furthermore, machine learning may offer a robust framework for integrating medical and imaging datasets, which may be beneficial for multifactorial and complicated cardiovascular disorders like heart failures
- In this study, we focus on new ML implementations in cardiovascular risk components, with a particular focus on cardiac imagery
- ML was found to be an excellent approach for predicting ACM in a comprehensive, prospective global analysis of individuals with suspicious CAD, outperforming clinically and CCTA factors independently
- Despite the fact that AI technologies in this sector are presently in their early stages of research and refining, the present quick growth in AI technologies in this domain might enable the frequent use of computerized CACS in medical practise in the coming years

The article "Machine Learning Approach for Cardiovascular Risk and Coronary Artery Calcification Score" was retracted in 2023. Reasons: signs of a paper mill; compromised peer review; unreliable results or conclusions.

## Figures and Tables

**Figure 1:** A single-layer neural network (NN) for machine learning against a deep neural network with four hidden layers.

**Figure 2:** Proposed flow chart for the machine learning analysis procedure for CAC.

**Figure 3:** Atherosclerotic vascular disorder prevalence by coronary artery calcium scoring classification. ASVD is an acronym for atherosclerotic vascular disorder.

**Figure 4:** The frequency distributions of coronary artery calcification (as measured by Agatston scoring) in RA patients and healthier regulate persons. The numbers across the bars represent the number of participants in every scoring subgroup as a percentage of the overall number of individuals.

**Figure 5:** The age-related incidence of coronary artery calcification in individuals with rheumatoid arthritis (RA) and healthy controls. For those under the age of 60, there was an important association among age and disorder conditions (*P* < 0.06 for interactions).

**Table 1:** The coronary calcification sampling (*n* = 470) compared to the overall ARIC Minneapolis and Forsyth County sampling in terms of age- and sex-adjusted variables (median or prevalent).

Parameters	Coronary artery calcification (CAC)	
	Median	Standard deviation
Carotid IMT (mm)	1.87	0.37
T. cholesterol (mg/dL)	323	51
HDL-C (mg/dL)	64	29
LDL-C (mg/dL)	245	47
Body mass index (kg/m^2^)	37.5	6.6
Triglycerides (mg/dL)	221	
Pack-years	25	20
Waist/hip ratio	1.02	0.19
Hypertension (%)	33	
Ever smoker (%)	67	
Diabetes (%)	6	

**Table 2:** Coronary artery calcification score clinical correlations.

	0	1-400	401-1000	>1000	*P* value
Preceding myocardial infarctions	7%	3%	11%	35%	<0.0002
Angina (%)	10%	12%	21%	52%	<0.0002
Recognized coronary artery disorders (%)	4%	20%	30%	64%	<0.0002
Any atherosclerotic vascular disorder	25%	34%	53%	90%	<0.0002

**Table 3:** Agatston calcium scores and the prevalence of coronary artery calcification in patients with initial and developed rheumatoid arthritis (RA) and healthy controls [46].

	Controller subjects (*n* = 97)	Initial RA (*n* = 80)	Recognized RA (*n* = 82)	Recognized vs. initial RA
Agatston score, average (IQR)	0 (0-20.3)	0 (0-53.7)	41.3 (0-459.9)	—
Prevalence of coronary-artery calcification (%)	49.48	53.97	71.67	
Agatston score subgroups (%)				
1 − 109	35.53	36.83	20.83	
>109	24.98	28.25	51.85	
OR (95% CI) unadjusted	1	2.32 (0.76-3.37)	4.04 (2.76-6.68)	3.62 (2.44-5.82)
*P*		0.66	<0.002	0.005
Adjusted for age and sex	1	2.42 (0.76-3.75)	3.84 (2.47-6.58)	3.09 (2.02-5.4)
*P*		0.56	0.006	0.059
Adjusted for cardiovascular risk factors	1	2.55 (0.78-4.20)	4.53 (2.66-8.64)	3.43 (2.06-6.24)
*P*		0.46	0.003	0.048

The article "Machine Learning Approach for Cardiovascular Risk and Coronary Artery Calcification Score" was retracted in 2023. Reasons: signs of a paper mill; compromised peer review; unreliable results or conclusions.

**Table 4:** Individuals with earlier and developed rheumatoid arthritis have different characteristics (RA).

Characteristics	Initial RA (*n* = 80)	Recognized (*n* = 82)	*P*
Rheumatoid element (%)	79.7	88.4	0.38
Number of swollen joints	4.0 (0.1-8.0)	5.0 (0.1-9.0)	0.86
C-reactive protein (mg/liter)	5.0 (4.1-11.1)	6.0 (4.1-27.0)	0.77
Erythrocyte sedimentation rate (mm/hour)	25 (6-35)	20 (8-53)	0.05
M-HAQ score	3.9 (2.3-6.1)	4.7 (2.8-6.7)	0.26
Pain VAS score	0.5 (0.1-0.7)	0.6 (0.2-2.0)	0.26
Disorder activity VAS score	3.0 (0.1-7.0)	3.0 (0.1-8.1)	0.99

## Data Availability

The data used to support the findings of this study are included within the article. Further data or information is available from the corresponding author upon request.
